The article "Identification of a miRSNP Regulatory Axis in Abdominal Aortic Aneurysm by a Network and Pathway-Based Integrative Analysis" was retracted in 2023. Reasons: signs of a paper mill; compromised peer review; unreliable results or conclusions.

# Identification of a miRSNP Regulatory Axis in Abdominal Aortic Aneurysm by a Network and Pathway-Based Integrative Analysis

**DOI:** 10.1155/2022/8776566

**Published:** 2022-10-13

**Authors:** Shenrong Liu, Yanfen Liao, Changsong Liu, Haobin Zhou, Gui Chen, Weiling Lu, Zheng Huang

**Affiliations:** ^1^Department of Cardiology, The First Affiliated Hospital of Guangzhou Medical University, Guangzhou, Guangdong 510120, China; ^2^Department of Stomatology, The Second People's Hospital of Panyu Guangzhou, Guangdong 511470, China; ^3^Department of Cardiology, The Second Affiliated Hospital, Army Medical University, Chongqing 400000, China; ^4^State Key Laboratory of Respiratory Disease, Department of Otolaryngology-Head and Neck Surgery, First Affiliated Hospital, Guangzhou Medical University, Guangzhou, Guangdong 510120, China; ^5^Department of Cardiology, Ganzhou Municipal Hospital, 49th, Grand Highway, 341000 Ganzhou, China

## Abstract

Abdominal aortic aneurysm (AAA) refers to local abnormal expansion of the abdominal aorta and mostly occurs in elderly men. MicroRNA (miRNA) is single-stranded RNA consisting of 18–25 nucleotides. It plays a key role in posttranscriptional gene expression and in the regulation of human functions and disease development. miRNA exerts its function mainly through the binding of complementary base pairs to the 3′ regulatory region of mRNA transcripts. Therefore, miRNA-related single-nucleotide polymorphisms (miRSNPs) can affect miRNA expression and processing kinetics. miRSNPs can be classified based on their location: miRSNPs within miRNA-producing genes and miRSNPs within miRNA target genes. Increasing evidence indicates that miRSNPs play an important role in the pathogenic kinetics of cardiovascular diseases. The aim of this study was to identify potential miRNAs and integrate them into a miRSNP-based disease-related pathway network, the results of which are of great significance to the interpretation of the potential mechanisms and functions of miRSNPs in the pathogenesis of diseases.

## 1. Introduction

Abdominal aortic aneurysm (AAA) represents a focal weakening and dilation of an inflammatory and degenerative abdominal aorta. It is the 15^th^ leading cause of death worldwide in individuals over 55 years [1]. Rupture is the most feared catastrophe of AAA with resultant 65%~85% mortality rate [2]. Currently, elective surgical remedy is only indicated once an aneurysm reaches 5.5 cm^3^, and the interventions for the vast majority of small but ongoing AAAs are clinically unproductive [3]. AAAs are results of complicated but poorly understood environmental and genetic risk factors, among which male gender and family history are substantial ones, suggesting a critical role of genetic components in AAA formation [4]. To date, a number of genetic studies have reported some AAA-specific risk alleles, however, with low odds ratio. The potent heritability of AAA and the low odds ratio of the risk alleles suggest that other genetic mechanisms underlying AAA remain to be explored.

The article "Identification of a miRSNP Regulatory Axis in Abdominal Aortic Aneurysm by a Network and Pathway-Based Integrative Analysis" was retracted in 2023. Reasons: signs of a paper mill; compromised peer review; unreliable results or conclusions.

MicroRNAs (miRNAs) are single-stranded 20-25 nucleotide RNA that are increasingly reported to be involved in the modulation of various biological and pathological processes [5, 6]. Notably, recent AAA studies have identified multiple miRNAs that participate in diverse key processes underlying AAA formation, including tissue inflammation, matrix degradation, cell proliferation and migration, and VSMC apoptosis [7–10]. More importantly, some miRNAs are validated to participate in the regulation of AAA onset and progression. For instance, inhibition of miR-188-5p could alleviate aortic matrix degradation, VSMC apoptosis, multiple inflammatory cell type infiltration, and decrease experimental murine AAA formation [11]; miR-126 could substantially reduce AAA formation by suppressing inflammatory cytokines generation and facilitating cell survival in mice [12]. This evidence indicates that miRNAs play important roles in AAA pathogenesis. A deeper understanding of the processes and regulations of miRNAs during AAA formation would favor a better comprehension and potential intervention strategy for AAA.

miRNAs have been well recognized to exert their functions mainly by transcriptionally regulating gene expression through binding to the specific target sites in the 3′-UTR of mRNA, which induces the translation suppression and degradation of mRNA [13]. Studies have suggested that since miRNAs are small molecules, any slight alterations in the sequence may potentially yield structural changes to alter their expression and interaction with target mRNAs, further tuning the expression level of the target genes [14–16]. Single-nucleotide polymorphisms (SNPs) are the polymorphisms in genes generated by variation of single nucleotide and are the most frequent form of human heritable variation. miRNA-associated SNPs (miRSNPs) are SNPs in genes encoding either miRNAs or the target transcripts of miRNA. It has been demonstrated that many miRSNPs can affect the expression and function of miRNAs by influencing the transcription and processing of miRNAs and by impacting the interaction between miRNAs and their target mRNAs, thus affecting the pathophysiological processes mediated by the miRNA target gene [17–21]. It has been corroborated that miRSNPs have significant roles in the pathogenesis of multiple diseases such as cardiovascular diseases, central nervous system disorders, myasthenia gravis, and a variety of cancers. For instance, rs662702 of the binding sites between miR-328 and 3'UTR of PAX6 mRNA significantly increased PAX6 levels and elevated the risk of epilepsy [22]. In AAA, a few studies have identified SNP rs5516 in KLK1 gene, rs764522 and rs1036095 of TGFBR2 gene, and s55945735 and rs353291 in miR145 that are associated with increased susceptibility to AAA [23, 24]. Meanwhile, given that a miRNA can bind to numerous mRNA transcripts and that a single mRNA target can be under the control of multiple miRNAs, delineating the network of miRSNPs in AAA formation may facilitate exploring potential physiopathological roles of miRSNPs in AAA and a more integrative comprehension of AAA pathogenesis.

The article "Identification of a miRSNP Regulatory Axis in Abdominal Aortic Aneurysm by a Network and Pathway-Based Integrative Analysis" was retracted in 2023. Reasons: signs of a paper mill; compromised peer review; unreliable results or conclusions.

In the current study, we aimed to construct a landscape of miRNPs potentially associated with AAA and elaborate a miRSNP-based AAA-related pathway network. Our findings may contribute to the interpretation of the potential mechanisms and functions of miRSNPs in the pathogenesis of AAA.

## 2. Materials and Methods

### 2.1. Analysis Software

R software (version number: 4.0.5) was used in this analysis, and Cytoscape software (version number: 3.8.2) was used to display the network diagram.

### 2.2. Collection of AAA Risk-Related Genes

We collected risk genes associated with AAA from PubMed (https://pubmed.ncbi.nlm.nih.gov/), NCBI-Gene (https://www.ncbi.nlm.nih.gov/gene), GeneCards (https://www.genecards.org/), and Phenolyzer (http://phenolyzer.wglab.org/). The search term was abdominal aortic aneurysm, the selected species was Homo sapiens, and the selected gene type was protein coding. The collected AAA risk-related genes were combined and used for further analysis.

### 2.3. Functional Enrichment Analysis of AAA Risk-Related Genes

To explore the functions of AAA risk-related genes, we performed Gene Ontology (GO) functional enrichment analysis and Kyoto Encyclopedia of Genes and Genomes (KEGG) enrichment analysis. The analysis was performed using the R software package ClusterProfiler. GO analysis includes 3 parts: biological process (BP), cellular component (CC), and molecular function (MF). To ensure the reliability of the enrichment results, we used the Benjamini-Hochberg false discovery rate (FDR) to correct the *P* value for multiple hypothesis tests. FDR < 0.05 indicated that an enrichment was significant.

### 2.4. Crosstalk Analysis between Pathways

We used the cumulative hypergeometric test to analyze the crosstalk between AAA risk gene-related pathways. The analysis was performed using the *phyper* function in R software. The specific parameters were phyper (*k* − 1, *M*, *NM*, *n*, and lower.tail = *F*), where *N* represents the total number of genes in the human genome, *M* represents the number of genes in one pathway, *n* represents the number of genes in another pathway, and *k* represents the genes involved in both pathways. The FDR was used to correct the *P* value for multiple hypothesis tests (P.adj < 0.05 indicated significance).

The article "Identification of a miRSNP Regulatory Axis in Abdominal Aortic Aneurysm by a Network and Pathway-Based Integrative Analysis" was retracted in 2023. Reasons: signs of a paper mill; compromised peer review; unreliable results or conclusions.

### 2.5. miRNA and miRNA Target Gene Datasets

We first downloaded all human miRNA data and sequences from MirBase (http://www.mirbase.org/) and then used the R software package BiomaRt to obtain the 3′UTR sequences of corresponding AAA risk-related genes for the prediction of miRNA-related target genes. We used 9 bioinformatics tools to predict miRNA target genes: miRanda, RNA22, TargetMiner, TargetScan, MirTarget2, PITA, PicTar, DIANA-microT, and miRmap. Among the 9 bioinformatics tools, miRNA targets that appeared in at least 7 tools were used for subsequent analyses. Next, we performed KEGG analysis of the target genes to identify the pathways of miRNA enrichment and used the Benjamini-Hochberg method to correct the *P* value (P.adj < 0.05 indicated significance).

### 2.6. Data Analysis of miRSNPs

miRSNPs included miRSNPs within miRNA genes and miRSNPs within miRNA target genes. We used PolymiRTS (https://compbio.uthsc.edu/miRSNP/, version 3.0), miRSNP (http://bioinfo.life.hust.edu.cn/miRSNP/, version 3.0), and MSDD (http://bio-bigdata.hrbmu.edu.cn/msdd/home.jsp, version 3.0) to predict the SNP sites of miRNAs. Then, we used PolymiRTS (version 3.0) and MSDD (http://bio-bigdata.hrbmu.edu.cn/msdd/home.jsp) and miRdSNPs (http://mirdsnp.ccr.buffalo.edu/) to predict the SNP sites of miRNA target genes and integrate the SNPs of miRNA target genes.

### 2.7. Construction of a Pathway-Based miRSNP Switching Network (PMSN)

We used the cumulative hypergeometric test to construct the PMSN. The analysis was performed using the *phyper* function in R software. The specific parameters were phyper (*k* − 1, *M*, *NM*, *n*, and lower.tail = *F*), where *N* is the total number of genes in the human genome, *M* is the number of genes in a pathway, *n* is the number of target genes in an miRNA, and *k* is the number of genes involved in both pathways and miRNA target genes. The FDR was also used to correct the *P* value for multiple hypothesis tests (P.adj < 0.05 indicated significance).

### 2.8. Identification and Characterization of Key Pathways and High-Risk Genes

To further investigate the regulatory role of miRNAs in key pathways, we generated schematic diagrams of key pathways from the KEGG database (https://www.genome.jp/kegg/) and obtained information on relevant risk genes encoding relevant protein complexes in the pathways. miRSNP-miRNA-mRNA-risk pathways were further characterized.

The article "Identification of a miRSNP Regulatory Axis in Abdominal Aortic Aneurysm by a Network and Pathway-Based Integrative Analysis" was retracted in 2023. Reasons: signs of a paper mill; compromised peer review; unreliable results or conclusions.

## 3. Results

### 3.1. Collection of AAA-Related Risk Gene

(1) We retrieved articles related to AAA from PubMed and collected genes. We then selected relevant genes that were significant in AAA association analyses. A total of 35 genes were included in the analysis (Table 1). (2) We collected AAA-related gens from NCBI-Gene; a total of 137 genes were selected. (3) We collected AAA risk-related genes from GeneCards and then selected the top 200 genes on the basis of relevance score. (4) We collected AAA-related genes from Phenolyzer and screened them by score. The top 200 genes were selected for further analyses. We deduplicated the above collected gene sets and obtained a total of 462 AAA risk-related genes (Supplementary Table 1) for subsequent analyses.

### 3.2. Functional Enrichment of AAA Risk-Related Genes

We performed GO and KEGG functional analyses of the 462 collected AAA risk-related genes. The GO analysis results indicated that the AAA risk-related genes were mainly enriched in extracellular matrix organization, epithelial cell proliferation, blood coagulation, hemostasis, and response to oxygen level. In the CC analysis, the AAA risk-related genes were mainly enriched in collagen-containing extracellular matrix, the endoplasmic reticulum lumen, and the vesicle lumen. In addition, MF was mainly enriched in extracellular matrix structural constituents, signaling receptor activator activity, and receptor ligand activity (Figure 1(a) and Supplementary Table 2). KEGG enrichment analysis indicated that AAA risk-related genes were mainly enriched in the AGE-RAGE signaling pathway in diabetic complications, human cytomegalovirus infection, proteoglycans in cancer, and the relaxin signaling pathway (Figure 1(b) and Supplementary Table 3).

### 3.3. Crosstalk between Pathways

To analyze the relationship between AAA-related pathways, we used the cumulative hypergeometric algorithm to construct crosstalk between pathways to form a pathway network. The results indicated that most of the pathways had significant interactions, such as human cytomegalovirus infection and lipid and atherosclerosis (Figure 2(a)). In addition, we found that human cytomegalovirus infection had the highest degree of connectivity among all pathways (Figure 2(b)).

### 3.4. Relationship between miRNAs and Target Genes

To analyze the relationship between miRNAs and target genes and obtain miRNA target gene pairs, we first obtained the annotation information for all human miRNAs from MirBase. Next, for the relevant risk genes, we used 9 bioinformatics tools to obtain miRNA-mRNA interactions and screened the interactions that appeared in at least 7 bioinformatics tools for subsequent analyses. The results indicated that a total of 1,403 miRNA target gene pairs were obtained (Supplementary Table 4).

The article "Identification of a miRSNP Regulatory Axis in Abdominal Aortic Aneurysm by a Network and Pathway-Based Integrative Analysis" was retracted in 2023. Reasons: signs of a paper mill; compromised peer review; unreliable results or conclusions.

We selected miRNAs with more than 12 miRNA target genes for display using a network diagram. There were a total of 34 miRNAs. The miRNAs with high connectivity included hsa-miR-93-3p, hsa-miR-106a-5p, has-miR-20a-5p, and hsa-miR-20b-5p (Figure 3). The target genes with high connectivity include ABCA1, TSC1, TGFBR2, and PTEN, indicating that these genes are more susceptible to miRNA regulation. In addition, we selected miRNAs with more than 12 target genes and performed KEGG analysis on their target genes to identify pathways that were enriched in miRNA target genes. A total of 34 miRNAs and their target genes were included in the analysis. The results indicated that the main pathways with enriched miRNA target genes were the AGE-RAGE signaling pathway in diabetic complications, the TGF-beta signaling pathway, proteoglycans in cancer, and protein digestion and absorption (Supplementary Table 5).

### 3.5. miRSNP Recognition

First, we studied the SNPs in miRNA genes. We predicted the SNPs of miRNAs from PolymiRTS and miRSNPs. The PolymiRTS analysis results indicated that 1 of the 34 miRNAs had SNP sites; the miRSNP analysis results indicated that 32 of the 34 miRNAs had SNP sites. The MSDD analysis results showed that 2 of the 34 miRNAs had SNP sites. We integrated the PolymiRTS, miRSNP, and MSDD results to obtain the SNP information for miRNAs, and a total of 169 miRNA-SNP variant pairs were obtained (Supplementary Table 6). Next, we analyzed the SNPs of miRNA target genes. The PolymiRTS analysis results showed that there were 55 SNPs of miRNA target genes; the MSDD analysis results indicated that there was 1 SNP of miRNA target genes; and the miRdSNP analysis results showed that there were 109 SNPs of miRNA target genes (Supplementary Table 7). We used network diagrams to show the relationship between miRNAs and the SNPs of their target genes. The results showed that the target genes corresponding to hsa-miR-29, hsa-miR-15, hsa-miR-497, and hsa-miR-195 had many SNP sites and that rs200966435, rs200713361, and rs77877520 controlled many miRNA target genes (Figure 4).

### 3.6. Construction of the PMSN

To better understand the relationship between SNPs of miRNA genes, SNPs of miRNA target genes, and pathways, we constructed a PMSN network (Figure 5(a)). There were 32 miRNAs with SNP sites in the large network, and all target genes corresponding to miRNAs had SNP sites. Next, we further analyze the PMSN network. We analyzed the pathway connectivity and found that the pathways with high connectivity were the AGE-RAGE signaling pathway in diabetic complications, human cytomegalovirus infection, proteoglycans in cancer, and the relaxin signaling pathway (Figure 5(b)), indicating that these pathways were susceptible to regulation by related miRNAs (Figure 5(c)). We analyzed the connectivity of miRNAs, and the results indicated that the connectivity of hsa-miR-16a/b, hsa-miR-19a/b-3p, and hsa-miR-15a/b was relatively high (Figure 5(d)) and that the degree of connectivity was 11 for most miRNAs (Figure 5(e)).

The article "Identification of a miRSNP Regulatory Axis in Abdominal Aortic Aneurysm by a Network and Pathway-Based Integrative Analysis" was retracted in 2023. Reasons: signs of a paper mill; compromised peer review; unreliable results or conclusions.

### 3.7. Identification and Characterization of Key Pathways and High-Risk Genes

Based on the above analysis, we found that the AGE-RAGE signaling pathway in diabetic complications is of great significance and is regulated by the most miRNAs. In addition, related studies have shown that diabetes can significantly increase the risk of various cardiovascular diseases, and several in-depth studies have addressed the relationship between diabetes and AAA [25–28]. Therefore, we further analyzed this pathway. We used a pathway map to visualize the collected AAA risk genes related to the AGE-RAGE signaling pathway in diabetic complications. A total of 64 related genes encode proteins or complexes in the AGE-RAGE signaling pathway in diabetic complications, of which 6 genes contain a miRSNP in the 3′UTR region (Figure 6(a)).

We further characterized the potential mechanism of the miRSNP-gene pathway to investigate the functions and pathways affected by miRSNPs. We found that F3, TGFBR1, TGFBR2, MAPK1, and PIK3R1 were substantially regulated by miRNAs. In addition, a total of 4 miRNA target gene pairs were verified experimentally. Furthermore, we found that the miRNA target genes not only affect the AGE-RAGE signaling pathway in diabetic complications but also may affect multiple pathways, including the MAPK signaling pathway and TGF-beta signaling pathway (Figure 6).

### 3.8. The Regulatory Role of miRNAs in Key Pathways

To further analyze these miRSNPs, we visualized the miRNAs associated with AAA risk genes in the AGE-RAGE signaling pathway in diabetic complications (Figure 7(a)). Because the relationships between miRNA, TGFBR1, and MAPK14 were experimentally verified, we focused on the effect of hsa-miR-20a-5p, hsa-miR-20b-5p, and hsa-miR-93-5p on the key gene F3. These miRNAs all share a common SNP site, namely, rs200713361. We further plotted 3′UTR base binding between 3 miRNAs and the target gene F3 (Figure 7(b)) to demonstrate that they have an important relationship; thus, we elucidated a potential mechanism: rs200713361 – F3 – hsa-miR-20-5p/hsa-miR-93-5p – AGE-RAGE signaling pathway in diabetic complications may have an important impact on AAA. We used miRSNPs as a breakthrough point and screened reliable miRSNP databases to reveal a regulation axis: “miRSNP-miRNA-mRNA-risk pathway.” We show, schematically, the effect of miRSNPs on AAA through gene regulation as well as pathway effects (Figure 8).

The article "Identification of a miRSNP Regulatory Axis in Abdominal Aortic Aneurysm by a Network and Pathway-Based Integrative Analysis" was retracted in 2023. Reasons: signs of a paper mill; compromised peer review; unreliable results or conclusions.

## 4. Discussion

In the current study, we screened a catalog of human risk genes associated with AAA formation, profiled the functional signaling pathways that enriches AAA, and identified miRNAs that possibly interact with and impact these pathways relevant to AAA risk. Further, by introducing miRSNPs as the genetic strategy and by using dependable miRSNP databases, we comprehensively compiled SNPs of the most possibly influential miRNA in AAA pathogenesis and further constructed a novel PMSN to depict a novel “miRSNP-miRNA-mRNA-risk signaling pathway” genetic pattern that may underlie AAA formation. Our results may advance the current knowledge of possible genetic mechanism of AAA and encourage future elaboration on the possible miRSNP-based involvement in AAA formation.

AAA is a complex vascular disorder with devastating consequence once ruptured. It is well recognized that genetic factors contribute substantially to the susceptibility of AAA. Previous twin studies reported an estimation of 70% heritability [29], and some have shown elevated propensity to AAA in first-degree relatives of the sufferers [30, 31]. In the current study, we screened 462 AAA risk-related genes and found they are mainly enriched in extracellular matrix organization, blood coagulation, hemostasis, and response to oxygen level, most of which are closely correlated with the typical pathology of an aneurysmal aorta [32]. Based on these genes, we identified the AAA risk pathways, including those related to the PI3K-AKT signaling pathway and AGE-RAGE signaling pathway in diabetic complications, which have been suggested to be involved in AAA formation by affecting aortic inflammation, oxidative stress, and VSMC proliferation and migration [33–35]. Of note, advanced glycation end products (AGE) and the receptors for AGE (RAGE) have been involved in the pathogenesis of numerous disorders, but its implication in AAA pathogenesis is recently understood.Cumulated data indicated that AGE − RAGE levels are elevated in the aortic tissue, skin, and plasma of AAA sufferers and that the activation of AGE − RAGE pathways can enhance the production of ROS and inflammatory cytokines that in turn incite the generation of MMPs; additionally, AGE − RAGE pathways can activate NF−*κ*B, a pivotal and potent transcription factor in AAA pathogenesis, thus altogether resulting in AAA formation [32]. We also identified other risk pathways related to human cytomegalovirus infection, proteoglycans in cancer, the relaxin signaling pathway, and so, which may also contribute to the pathogenesis of AAA. These results are in align with the previous data showing that cytomegalovirus was more frequently detected in the plasma of AAA sufferers than in healthy controls and that its infection is associated with local aortic inflammation and more rapid aneurysmal clinical progression [36, 37]. Additionally, the risk of cancer was significantly increased in AAA patients compared to control, and cancer was one of the top causes of death in AAA cohorts. Thus, our findings help to inform the possibly important roles of several signaling pathways once atypical to AAA formation and may underscore a potential interrelationship between AAA and some other diseases, which may facilitate a more comprehensive understanding the how AAA evolves and progresses.

The article "Identification of a miRSNP Regulatory Axis in Abdominal Aortic Aneurysm by a Network and Pathway-Based Integrative Analysis" was retracted in 2023. Reasons: signs of a paper mill; compromised peer review; unreliable results or conclusions.

As one of the paradigmatic subjects of RNA interference, miRNAs have been recognized as potent participants in multiple pathological pathways and processes, and the dysregulation of miRNAs is tightly involved in the pathogenesis of various diseases [38], AAA included. To identify the potential functional miRNAs in AAA formation, we used reliable miRNA bioinformatics tools and retrieved a total of 1403 miRNA target pairs. Given that a single miRNA is capable of binding diverse target mRNAs, we further selected miRNAs with more than 12 miRNA target genes and built a network based on the 34 identified miRNAs. These miRNAs may thus have larger potential as crucial regulatory nodes in AAA-associated risk pathways. A further pathway network based on these miRNAs were build, and we found several miRNAs with high connectivity such as miR-29, miR-let7 family, and miR-16, some of which are demonstrated to influence AAA formation by experimental evidences. For instance, it has been reported that miRNA let-7a could influence the proinflammatory IL-6 by acting as an endogenous competing RNA that targets IL-6 mRNA to impact the AAA progression in mice [39]. We also found that those miRNAs with high connectivity also tend to have high connectivity in PMSN and have more SNPs in their encoding genes, such as hsa-miR-29, hsa-miR-15, and hsa-miR-497. However, due to insufficient emerging experimental evidence on the relationship between miRSNPs and diseases, our results are not experimentally echoed. Thus, these findings should be regarded as notion-innovative and be interpreted with caution.

Then, we explored the miRSNPs that may be associated with AAA formation. We focused on studying miRSNPs instead of SNPs of protein-encoding genes in view of several reasons. First, there are much scarcer SNPs identified hitherto in protein-encoding genes than in noncoding regions such as miRNA-encoding genes [40], so miRSNP detection may be more effective and economic as target-identification strategy. Second, due to the much smaller size of miRNA compared with protein-encoding genes, SNPs can exist solely in miRNA-encoding genes but not in protein-encoding genes. Multiple SNPs in protein-encoding genes can substantially increase the possibility of SNPs to work oppositely to cause neutralized and weaker integrated biological potency. As for miRNAs, due to their short sequence, any slight alterations caused by SNPs may potentially yield structural changes that alters the expression of miRNAs and their interaction with targets [14, 15, 41]. Third, given the diversity of intracellular regulation mediators of proteins in contrast to miRNAs, the interference of one SNP on gene expression may be modest during the whole cellular journey for proteins [41]. We further constructed the PMSN to assess the underlying impact of miRSNPs on AAA susceptibility at a pathway level  [42] .Notably, the major signaling pathways based on our PMSN largely overlapped with the major ones derived from AAA risk genes (such as AGE − RAGE signaling pathway in diabetic complications, human cytomegalovirus infection, PI3K − Akt pathways, and the relaxin signaling pathway), with even higher degree of connectivity of the pathways, suggesting the validity and even higher potency of miRSNP − based identification strategy.Thus, the novel miRSNP − based strategy is of large potential in identifying underlying pathways and targets and a deeper comprehension of the pathogenesis of diseases including AAA.Meanwhile, some has suggested that PMSN may also facilitate recognition of different and even irrelevant molecular processes and identification of signaling pathways underlying the pathology in diseases of similar types [43]. Taken together, our identified rs200713361 − F3 − hsa − miR − 20 − 5p/hsa − miR − 93 − 5p − AGE − RAGE signaling pathway may have significant roles in the pathogenesis of AAA and even some diseases with similar pathology (such as thoracic aortic aneurysm), which merits future investigation and extrapolation.

The article "Identification of a miRSNP Regulatory Axis in Abdominal Aortic Aneurysm by a Network and Pathway-Based Integrative Analysis" was retracted in 2023. Reasons: signs of a paper mill; compromised peer review; unreliable results or conclusions.

Interestingly, some previous studies have suggested an evidently low absolute frequency of SNPs located in miRNAs [43]; nonetheless, our analysis on miRSNP showed that 32 out of 34 selected miRNAs with more than 12 potential targets have a total of 169 SNPs in their coding genes, with a large proportion of the miRNAs share some common polymorphisms. One of the suppositions derived from this finding is that it is the abundant SNPs in the miRNA-encoding genes that is one of the underlying mechanisms for the diversity of downstream targets of these miRNAs, given the short sequence of miRNA that may readily undergo an easier change in structure and function by single-nucleotide variation. Accordingly, one might further infer that combining abundant SNP-associated strategy may help improve the efficacy in identification of miRNAs that possess multiple functional targets and have potentially potent biological regulation in disease development.

There are certain limitations in our study. First, we selectively chose miRNAs with more than 12 known target genes for further analysis and PMSN construction. It should be noticed that the miRNAs filtered out may also have primary impact on AAA pathogenesis and that our analysis may have underestimated the scope of effect of miRNAs and miRSNPs on AAA formation. Nonetheless, we found that the most significant KEGG pathways deduced from our miRNA-based PMSN overlapped substantially with those derived from AAA risk genes, suggesting that the filtered miRNAs should be representative of the major functionally active miRNAs in AAA pathophysiology. Second, while causality do has been established between certain miRSNPs and some diseases, a caution should be mentioned that most SNPs identified to date are not functionally valid [44], and even when valid, they are incapable of causing final biological consequences due to multiple confounding intracellular regulation factors. Thus, the existence and potency of the regulation and function of miRSNPs in AAA formation suggested by our PMSN merit concrete and definitive experimental verification in the future.

In conclusion, the current study explored the possible participation of miRSNPs in AAA pathogenesis. For the first time, we constructed a novel PMSN to depict a novel “miRSNP-miRNA-mRNA-risk signaling pathway” genetic pattern that may underlie AAA formation. Our results contribute to a deeper comprehension of possible genetic mechanism underlying AAA and encourage future elaboration on the possible miRSNPs-based involvement in AAA formation.

## Figures and Tables

**Figure 1:** Functional enrichment analysis of AAA risk-related genes. (a) GO functional enrichment analysis of AAA-related genes; the color indicates -Log10 (FDR), and the more red is the color, the more significant is the enrichment; the circle indicates BP, the triangle indicates the CC, the square indicates the MF, and the shape size indicates the number of enriched genes. The larger is the shape, the greater is the number of enriched genes. (b) The relationship between genes and pathways. The left semicircle indicates the genes, the right semicircle indicates the pathways to which the genes are enriched, and the color indicates different pathways. BP: biological process; CC: cellular component; MF: molecular function.

The article "Identification of a miRSNP Regulatory Axis in Abdominal Aortic Aneurysm by a Network and Pathway-Based Integrative Analysis" was retracted in 2023. Reasons: signs of a paper mill; compromised peer review; unreliable results or conclusions.

**Figure 2:** Crosstalk between AAA-related pathways. (a) We analyzed the path crosstalk network using the cumulative hypergeometric algorithm. The size of the dot represents the degree of connectivity of the pathways, and the larger is the shape, the higher is the degree of connectivity; the connection line represents the relationship between the paths, and a darker color indicates a more significant relationship between pathways. (b) The histogram represents the distribution of the connectivity of the pathways. The horizontal axis is connectivity, and the vertical axis is the pathway.

**Figure 3:** The relationship between miRNAs and target genes. (a) Network diagram showing the relationship between miRNAs and target genes. Pink indicates miRNA, and blue indicates miRNA target genes. The size of the shape indicates the degree of connectivity (the larger is the shape, the higher is the degree of connectivity). (b) Network diagram showing the relationship between miRNAs and pathways with enriched target genes. Blue represents miRNA, and orange represents the KEGG pathway. The size of the shape indicates the degree of connectivity; the larger is the shape, the higher is the degree of connectivity. The thickness of the line indicates the degree of enrichment; the thicker is the line, the more enrichment of the miRNA target gene in the pathway.

**Figure 4:** Network diagram showing the relationship between miRNAs and the SNPs of their target gene. Pink represents miRNAs, and blue represents the SNPs in the miRNA target genes. The larger is the shape, the higher is the degree of connectivity.

**Figure 5:** PMSN analysis. (a) The construction of the PMSN network. Orange represents the KEGG pathway; blue represents miRNA. The node size represents the degree of connectivity, and larger nodes indicate higher connectivity. The red circle indicates that the miRNA had no SNP site. The connecting line between miRNA and pathways indicates that there is a relationship between the miRNA and the pathway, and a red connecting line indicates that the miRNA target gene has SNPs. The thickness of the connecting line represents the adjusted *P* value. (b) The histogram shows the top 10 pathways. (c) Histogram of the distribution of pathway connectivity. (d) Histogram of the top 10 miRNAs in terms of degree of connectivity. (e) Histogram of the distribution of miRNAs.

**Figure 6:** The effect of AAA risk genes on the AGE-RAGE signaling pathway in diabetic complications in the KEGG database. (a) Boxes with red outlining indicate proteins or related complexes encoded by AAA risk-related genes, and boxes surrounded by orange indicate that the corresponding coding gene contains a miRSNP in the 3′-UTR. (b) Schematic diagram of the miRSNP-miRNA-gene-pathway axis. The yellow ellipse indicates a risk gene, the blue ellipse indicates miRNA, and the red five-pointed star indicates that the miRNA target relationship has been experimentally verified. We marked the SNP of the target gene on line between the miRNA and the risk gene. A red outer circle represents the pathway, green represents the AGE-RAGE signaling pathway in diabetic complications, and blue represents the TGF-beta signaling pathway.

The article "Identification of a miRSNP Regulatory Axis in Abdominal Aortic Aneurysm by a Network and Pathway-Based Integrative Analysis" was retracted in 2023. Reasons: signs of a paper mill; compromised peer review; unreliable results or conclusions.

**Figure 7:** Effect of miRNA on the AGE-RAGE signaling pathway in diabetic complications. (a) Red font indicates the protein or complex encoded by miRNA target genes. (b) The schematic diagram illustrates the potential mechanism underlying the effect of hsa-miR-20a-5p, hsa-miR-20b-5p, and hsa-miR-93-5p on the F3 gene. The gene may play an important role in AAA through the rs200713361 mutation site.

**Figure 8:** A model illustrating the effect of miRSNP-miRNA-mRNA-risk signaling pathway on AAA.

**Table 1:** Candidate genes highly associated with AAA in association analyses from relevant literature review retrieved from PubMed.

Gene	Sample	Result	PUBMEDID
PCSK9	7,642 European ancestry cases, 172,172 European ancestry controls	rs11591147,p-value=6e-11,OR=1.58	32981348
LPA	7,642 European ancestry cases, 172,172 European ancestry controls	rs118039278,p-value=4e-18,OR=1.28	32981348
CHRNA3	7,642 European ancestry cases, 172,172 European ancestry controls	rs55958997,p-value=9e-14,OR=1.12	32981348
ABHD16B	7,642 European ancestry cases, 172,172 European ancestry controls	rs73149487,p-value=8e-09,OR=1.26	32981348
GDF7	7,642 European ancestry cases, 172,172 European ancestry controls	rs7255,p-value=9e-13,OR=1.1	32981348
MEPE	7,642 European ancestry cases, 172,172 European ancestry controls	rs10023907,p-value=2e-08,OR=1.09	32981348
CDKN1A	7,642 European ancestry cases, 172,172 European ancestry controls	rs3176336,p-value=1e-10,OR=1.1	32981348
TRIB1	7,642 European ancestry cases, 172,172 European ancestry controls	rs10808546,p-value=1e-10,OR=1.1	32981348
LIPA	7,642 European ancestry cases, 172,172 European ancestry controls	rs1412445,p-value=1e-10,OR=1.1	32981348
ZPR1	7,642 European ancestry cases, 172,172 European ancestry controls	rs964184,p-value=5e-19,OR=1.18	32981348
APOA5	7,642 European ancestry cases, 172,172 European ancestry controls	rs964184,p-value=5e-19,OR=1.18	32981348
ADAMTS8	7,642 European ancestry cases, 172,172 European ancestry controls	rs4936098,p-value=7e-16,OR=1.13	32981348
CRISPLD2	7,642 European ancestry cases, 172,172 European ancestry controls	rs35254673,p-value=3e-08,OR=1.09	32981348
CTAGE1	7,642 European ancestry cases, 172,172 European ancestry controls	rs4401144,p-value=4e-14,OR=1.11	32981348
APOE	7,642 European ancestry cases, 172,172 European ancestry controls	rs429358,p-value=1e-15,OR=1.17	32981348
LDLR	1,755 European ancestry cases, 5,314 European ancestry controls	rs6511720,p-value=2e-10,OR=1.32	24046328
LRP1	1,737 European ancestry cases, 5,435 European ancestry controls,129 cases	rs1466535,p-value=5e-10,OR=1.15	22055160
RBBP8	1,516 European ancestry intracranial aneurysm cases, 818 European ancestry abdominal aortic aneurysm cases, 760 European ancestry thoracic aortic aneurysm cases, 9,507 European ancestry controls	rs8087799,p-value=2e-09,OR=1.21	27418160
ANKRD44	1,516 European ancestry intracranial aneurysm cases, 818 European ancestry abdominal aortic aneurysm cases, 760 European ancestry thoracic aortic aneurysm cases, 9,507 European ancestry controls	rs919433,p-value=5e-08,OR=1.18	27418160
CELSR2	4,972 European ancestry cases, 99,858 European ancestry controls	rs602633,p-value=7e-09,OR=1.14	27899403
PSRC1	4,972 European ancestry cases, 99,858 European ancestry controls	rs602633,p-value=7e-09,OR=1.14	27899403
SORT1	4,972 European ancestry cases, 99,858 European ancestry controls	rs602633,p-value=7e-09,OR=1.14	27899403
IL6R	4,972 European ancestry cases, 99,858 European ancestry controls	rs12133641,p-value=5e-13,OR=1.14	27899403
CDKN2B-	4,972 European ancestry cases, 99,858 European ancestry controls	rs10757274,p-value=2e-33,OR=1.24	27899403
DAB2IP	4,972 European ancestry cases, 99,858 European ancestry controls	rs10985349,p-value=2e-11,OR=1.171	27899403
SMYD2	4,972 European ancestry cases, 99,858 European ancestry controls	rs1795061,p-value=9e-11,OR=1.131	27899403
LINC00540	4,972 European ancestry cases, 99,858 European ancestry controls	rs9316871,p-value=5e-10,OR=1.15	27899403
ZNF335	4,972 European ancestry cases, 99,858 European ancestry controls	rs58749629,p-value=2e-17,OR=1.223	27899403
PCIF1	4,972 European ancestry cases, 99,858 European ancestry controls	rs58749629,p-value=2e-17,OR=1.223	27899403
MMP9	4,972 European ancestry cases, 99,858 European ancestry controls	rs58749629,p-value=2e-17,OR=1.223	27899403
ERG	4,972 European ancestry cases, 99,858 European ancestry controls	rs2836411,p-value=6e-09,OR=1.113	27899403
FERMT1	4,972 European ancestry cases, 99,858 European ancestry controls	rs6516091,p-value=3e-06,OR=1.131	27899403
LDAH	4,972 European ancestry cases, 99,858 European ancestry controls	rs13382862,p-value=1e-06,OR=1.1	27899403
CDKN2A	1,292 European ancestry cases, 30,503 European ancestry controls	rs2383207,p-value=2e-08,OR=1.27	20622881
CDKN2B	1,292 European ancestry cases, 30,503 European ancestry controls	rs2383207,p-value=2e-08,OR=1.27	20622881

The article "Identification of a miRSNP Regulatory Axis in Abdominal Aortic Aneurysm by a Network and Pathway-Based Integrative Analysis" was retracted in 2023. Reasons: signs of a paper mill; compromised peer review; unreliable results or conclusions.

## Data Availability

The data used to support the findings of this study are included within the article.

## Supplementary Materials

Supplementary 1 Supplementary Table 1: four hundred and sixty-two candidate genes highly associated with AAA according to the combination of PubMed, NCBI-Gene, GeneCards, and Phenolyzer.

Supplementary 2 Supplementary Table 2: Gene Ontology analysis of the 462 candidate AAA risk-related genes.

Supplementary 3 Supplementary Table 3: KEGG enrichment analysis of the 462 candidate AAA risk-related genes.

Supplementary 4 Supplementary Table 4: bioinformatic prediction on miRNA-mRNA interactions based on the 462 candidate AAA risk-related genes and human miRNAs.

Supplementary 5 Supplementary Table 5: KEGG enrichment analysis of 34 miRNAs (with more than 12 target genes) and their target genes.

Supplementary 6 Supplementary Table 6: predicted miRNA-SNP variant pairs based on PolymiRTS, miRSNPs, and MSDD databases.

Supplementary 7 Supplementary Table 7: predicted SNPs of miRNA target genes and their paired miRNAs based on PolymiRTS, miRSNPs, and MSDD databases.
